# GIS Multimedia Technology in Regional Construction Land Suitability Evaluation in Mountainous Villages and Towns

This article has been retracted.

**DOI:** 10.1155/2022/8305285

**Published:** 2022-06-26

**Authors:** Zhenhong Zhou, Huihui Wang, Qi Hu, Min Zhou

**Affiliations:** School of Forestry and Landscape Architecture, Anhui Agricultural University, Hefei, Anhui 230036, China

## Abstract

In order to explore the suitability evaluation of regional construction land in mountainous villages and towns, a method based on GIS technology is proposed. Supported by GIS and RS technology, the Delphi method is used to determine the natural, socioeconomic, and ecological security factors affecting the ecological suitability of regional construction land in mountainous villages and towns, and analytic hierarchy process is used to calculate the weight of relevant influencing factors. Following the principle of giving priority to ecological protection, a set of ecological suitability evaluation model system and method of regional construction land in mountainous villages and towns are established, based on which the basic ecological control areas of mountainous villages and towns in the study area are divided, so as to provide suggestions for rational and effective planning of land resources in mountainous villages and towns. The experimental results show that the K-means clustering method is divided into five categories: the most suitable land, the more suitable land, the basically suitable land, the unsuitable land, and the unavailable land. Finally, according to the suitability grade system of construction land, it is reclassified, the unsuitable land and unavailable land are divided into basic ecological control areas, the most suitable land and more suitable land are divided into construction control areas, and the basically suitable land is listed as ecological buffer areas. It is proved that the basic ecological control area determined by the model method is basically consistent with the current basic ecological control line of a city, which shows that the model is practical and scientific.

## 1. Introduction

Therefore, we must put forward scientific, rational, and sustainable land-use methods and measures [1]. The research on the regional construction land conditions of mountainous villages and towns can provide a scientific basis for the strategic decision-making of regional sustainable development of mountainous villages and towns. It involves many aspects such as nature, society, economy, environment, land, engineering, and so on. It is a complex systematic project. Its decision-making results play an important role in cherishing and making rational use of land and protecting land resources around mountainous villages and towns. The previous research methods of land use for regional development of mountainous villages and towns are generally evaluated and planned by the staff who have been engaged in the regional planning of mountainous villages and towns for a long time through field investigation, and then combined with the method of empirical analysis. This conventional method has a large amount of investigation workload, difficult unified standards, poor spatial positioning accuracy, certain subjective randomness, and is not easy to carry out quantitative research. The idea and method of geographic information system (GIS) are helpful to combine the investigation of regional land conditions in mountainous villages and towns with database management, the implementation of planned land evaluation with spatial analysis method, and the decision-making of regional layout with the design of application model base, so as to enhance the ability of spatial analysis and real-time update, It improves the spatial decision-making level of regional land-use management in mountainous villages and towns, especially for the research on land use decision-making of multiobjective and multifactor regional development planning in mountainous villages and towns, which has extensive and potential advantages [2]. It realizes the quantification, standardization, standardization, systematization, and informatization of ecological suitability evaluation of regional construction land in villages and towns and will become an important topic for scientific urban planning.

Villages and towns are the link between urban economy and rural economy, and the radiation scope is the vast rural areas. The purpose is to occupy a lot of land resources, especially cultivated land resources, in the regional construction of local villages and towns. The land use is extensive, and the per capita cultivated land area is lower than the minimum survival guarantee line (0.8 mu) proposed by FAO. The regional land problem of villages and towns is a major problem at present. Today, with population growth, population aging, and serious environmental damage, it is more necessary to use land reasonably, protect cultivated land, improve land utilization and productivity, and maintain and improve the ecological function of land [3]. The impact of natural ecological environment conditions on the regional construction of villages and towns is multifaceted, such as the restriction of topographic conditions will affect the development scale and land layout of villages and towns. Engineering geology, hydrogeology, and special gas edge conditions will affect the selection, scale, layout, and construction of specific projects in local villages and towns. The ecological suitability evaluation of construction land in villages and towns is to evaluate the quality of the environmental conditions of the land according to the needs of planning and construction, based on the investigation, collection, and analysis of the data of natural environmental factors, so as to determine the applicability of the land to the regional construction use of villages and towns, and provide a scientific basis for the rational selection and layout of construction land in villages and towns [4]. The ecological suitability evaluation method of regional construction land in villages and towns mainly adopts the natural ecological planning method and takes the suitability evaluation of regional construction land in villages and towns as the research object. Through the analysis of natural attribute factors of regional land use in villages and towns and the research of GIS integration technology, the theories and methods of system science, mathematics, computer science, urban planning, ecology, and other disciplines are comprehensively applied. The purpose is to establish the ecological suitability evaluation of regional construction land in mountainous villages and towns. Based on the investigation and analysis of the natural and socioeconomic conditions of mountainous villages and towns, a comprehensive and comprehensive quality evaluation is carried out according to the requirements of ecological protection and construction, so as to determine the suitability of land [5]. Liu et al. [6] used the multifactor comprehensive evaluation method to evaluate and analyze the suitability of unused land [6]. Xiao et al. [7] used Arc View software to build a planting suitability evaluation system to evaluate characteristic cash crops [7]; Mishra et al. [8] takes GIS as the system environment, simulates the geospatial process through cellular automata, determines the conversion rules between cellular neighborhoods through “niche,” constructs the cellular automata niche suitability model, and obtains the hierarchical map of the suitability of land development and construction on low hills and gentle slopes [8].

Based on this, this paper uses Delphi method to determine the natural, socioeconomic, and ecological security factors affecting the ecological suitability of mountain village and town regional construction land, uses analytic hierarchy process to calculate the weight of relevant influencing factors, and establishes a set of ecological suitability evaluation model system and method of mountain village and town regional construction land. Based on this, the basic ecological control areas of mountainous villages and towns in the study area are divided, and the suggestions on regional land use of mountainous villages and towns are put forward from the perspective of protecting the regional ecological environment of mountainous villages and towns, so as to provide a useful attempt and supplement for the regional development of mountainous villages and towns.

## 2. Evaluation Principle and System

### 2.1. Evaluation Principles

In the process of suitability evaluation, the selection and standardization of indicators, the determination of weight, and how to combine GIS with decision-making process are always the key to the research of evaluation methods. Taking the ecological suitability evaluation of regional construction land in mountainous villages and towns as the main research object, this paper determines the following evaluation principles: (1) the principle of ecological priority. If an area is found to have important ecological value, this factor has the priority to decide, and the development of such areas is strictly limited; (2) comprehensive principle determines the index system according to the comprehensive characteristics of land use in mountainous villages and towns and pays attention to the comprehensiveness and representativeness of the index; (3) according to the principle of adjusting measures to local conditions, the selected factors should be coordinated with the regional data and technical level, and the data closest to the land use status and better reality of the study area should be used for evaluation [9].

### 2.2. Evaluation System

This paper comprehensively considers the development objectives of mountainous villages and towns in the study area, the current land use situation of mountainous villages and towns, and the problems in the current regional construction of mountainous villages and towns, and finally establishes an index evaluation system in line with this study under the guidance of ecological suitability evaluation theory, following the principle of ecological priority and according to the hierarchical relationship between indicators. The influencing factors of ecological suitability of regional construction land in mountainous villages and towns are divided into natural factors, socioeconomic factors, and ecological security factors [10]. First, the vegetation and landscape distribution in the study area are investigated from the perspective of protecting the ecology and socioeconomic security of mountainous villages and towns, so as to obtain the regional scope with ecological protection value and historical and cultural value, such as basic farmland protection, nature reserve, protected water area, cultural landscape. Second, the selection of evaluation indicators is considered from the natural factors, including topography, geology, water area, vegetation and other factors. Third, the selection of evaluation indicators is considered from socioeconomic factors, including land use status, built-up areas, traffic location advantages, and so on. According to the above evaluation principles and index analysis, the ecological suitability evaluation index system is composed of 16 single factors in three aspects: natural factors, socioeconomic factors, and ecological security factors (Figure 1), in which *A* is the target layer, *B* is the middle layer, and *C* is the index layer.

## 3. Evaluation Model and Method

### 3.1. Suitability Evaluation Model

The multifactor comprehensive evaluation model is used to evaluate the comprehensive suitability of each factor. This paper proposes the suitability evaluation model of regional construction land in mountainous villages and towns as follows:

(1) $$\begin{array}{c} S=\sum_{i=1}^{n}B_{i}W_{i}, \end{array}$$

where *S* is the comprehensive evaluation index of ecological suitability; *B*_*i*_ is the score of the *i*-th evaluation factor (dimensionless); *W*_*i*_ is the weight of the *i*-th evaluation factor; and *n* is the number of factors participating in the evaluation.

### 3.2. Evaluation Grade of Construction Land

The evaluation of regional construction land in mountainous villages and towns is usually based on the ecological protection measures determined by the natural conditions, socioeconomic conditions, and local laws and regulations of the construction land, and combined with the construction requirements. According to the degree of ecological suitability of construction land, it is divided into five levels: most suitable, more suitable, basically suitable, unsuitable, and unavailable land (Table 1) [11]. The unsuitable land and unavailable land shall be classified as the basic ecological control area, and all construction activities shall be prohibited in this area to ensure ecological security. The most suitable land and more suitable land are classified as the construction control area, and the construction land generally cannot exceed this area. The basically suitable land is divided into ecological buffer area for the isolation of basic ecological control area and construction control area to ensure a buffer space between them.

### 3.3. Index Quantitative Classification Standard

After the evaluation factors are determined, the natural and socioeconomic conditions of the study area shall be comprehensively investigated and repeatedly demonstrated. According to the influence degree of each evaluation factor on the regional construction land of mountainous villages and towns, it is divided into multiple ecological suitability grades. In this paper, the suitability evaluation value of evaluation factors is determined as grade 5, and 5, 4, 3, 2 and 1 represent the ecological suitability score of evaluation factors.

### 3.4. Determination Method of Evaluation Index Weight

In order to ensure the scientificity and accuracy of the weight of evaluation factors, the analytic hierarchy process is used to compare and judge the relative importance of indicators at all levels, maintain the consistency of judgment matrix, and finally obtain the weight value of each indicator [4].

#### 3.4.1. Principle of Determining Weight

① Establish a hierarchical structure model, analyze the relationship between indicators, and build a multilevel index system (Figure 1). The hierarchy is generally divided into target layer, which has only one element, which is generally the predetermined goal and ideal result of analyzing the problem; The criterion layer includes the intermediate links involved in achieving the goal. It is composed of several levels, including the criteria and subcriteria to be considered, index level, including various measures and decision-making schemes available for achieving objectives.
② Construction of comparison judgment matrix *A*
The indicators at the same level are compared in pairs for a certain factor at the upper level. Determine the quantitative scale method of thinking judgment, and use the scale of importance 1 ∼ 9. *a*_*ij*_ generally takes the scale of 1, 3, 5, 7, and 9. Its meaning is: 1 indicates that the two elements have the same importance, 3 indicates that the former is slightly important, 5 indicates that the former is obviously important, 7 indicates that the former is strongly important, and 9 indicates that the former is extremely important; and 2, 4, 6, and 8 are the intermediate values of the above judgment [12].
  (2) $$\begin{array}{c} A=\left[\begin{array}{cccc} a_{11} & a_{12} & ... & a_{1n}\\ a_{21} & a_{22} & ... & a_{21n}\\ ... & ... & ... & ...\\ a_{m1} & a_{m1} & ... & a_{mn} \end{array}\right]. \end{array}$$
Obviously, the judgment matrix must meet
  (3) $$\begin{array}{c} \left\{\begin{array}{cc} a_{ij}=\frac{1}{a_{ij}}=\frac{W_{i}}{W_{j}\left(i\neq j\right)}, & \left(i,j=1,2,\ldots ,n\right),\\ a_{ij}=1, & \left(i=j\right). \end{array}\right. \end{array}$$
③ Hierarchical single sorting
For the judgment matrix *A*, the calculation satisfies *AW*=*λ*_max_*W* (*λ*_max_ is the maximum eigenvalue of *A*, *W* is the normalized eigenvector corresponding to *λ*_max_, and the component *W*_*i*_ of *W*: is the weight value of single ranking of corresponding elements). The root square method is used to solve the normalized eigenvector and eigenvalue, that is, first calculate the *n*-th root W¯i=Min of the product of each row scale of the judgment matrix (*M*_*i*_=∏_*j*=1_^*n*^*a*_*ij*_ is the value of each row element of the judgment matrix). Normalize the square root vector to obtain the *i*-th component $W_{i}=\sum_{i=1}^{n}{\bar{W}}_{i}/{\bar{W}}_{i},\;\left(i=1,2,\ldots ,n\right)$ of the eigenvector *W*. Finally, calculate the maximum eigenvalue *λ*_max_=∑_*i*=1_^*n*^(*AW*)/(*nW*_*i*_) of the judgment matrix ((*AW*)_*i*_ is the *i*-th component of vector *AW*). In order to test the consistency of the judgment matrix, it is necessary to calculate its consistency index: CI=*λ*_max_ − *n*/*n* − 1, and compare CI with the average random consistency index RI (Figure 2), which is recorded as CR. When CR=CI/RI < 0.10, the judgment matrix is considered to have satisfactory consistency [13].
④ Hierarchical total sorting

Using the results of single-level sorting, the weight of the importance of all elements in this level relative to the previous level can be calculated, that is, the total level sorting. Check the consistency of the hierarchical total ranking results. When the consistency index meets the standard, it is considered that the hierarchical total ranking results are acceptable [14].

(4) $$\begin{array}{c} B_{n}=\sum_{j=1}^{m}a_{j}b_{n}^{j}, \end{array}$$

where *B*_*n*_ is the weight of the index layer, *a*_*j*_ is the weight of each factor of the criterion layer relative to the target layer, and *b*_*n*_^*j*^ is the weight of each factor of the index layer relative to the criterion layer. Obviously,

(5) $$\begin{array}{c} \sum_{i=1}^{n}\sum_{j=1}^{m}a,b_{i}^{j}=1. \end{array}$$

Total sorting consistency formula is as follows:

(6) $$\begin{array}{c} \text{CR}=\frac{\sum_{j=1}^{m}\left|a_{j}{\text{CI}}_{j}\right|}{\sum_{j=1}^{m}\left(a_{j}{\text{RI}}_{j}\right)}. \end{array}$$

When CR < 0.10, it is considered that the ranking has satisfactory consistency, that is, the weight of the evaluation index is obtained.

#### 3.4.2. Determination of Weight

The weight of each primary index and secondary index in the evaluation system is gradually calculated by using analytic hierarchy process (Table 2).

## 4. Case Analysis

A city is located in the Pearl River Delta with rapid economic development. The city has a land area of 1952.84 kmz and a coastline of 260 km. The area is high in the southeast and low in the northwest, most of which are low mountains and hills, with flat platforms in the middle and coastal plains in the West. The index system and evaluation model are used to evaluate the ecological suitability of construction land in a city, and the basic ecological control area of a city is extracted according to the evaluation results [1]. The TM remote-sensing image is processed by PCI remote-sensing image software, and the evaluation factor information of vegetation, water area, built-up area, and road in the study area is obtained through multiband image fusion, correction, registration, and visual interpretation. Use ArcGIS software to obtain land-use type information such as industry and mining, residential land, dry land, grassland and forest land from the current land use map, and extract evaluation index information such as elevation, slope, aspect, and geomorphic type from the 1 : 250000 topographic map [15]. Using relevant maps and data, we can get the information of foundation bearing capacity, protected areas, cultural landscapes, protected water areas, basic farmland protection, and so on. With the support of ArcGIS, it is transformed into a projection coordinate system consistent with the national l : 250000 basic terrain database, and the layer is transformed into grid format. The grid size is 50 m × 50 m, which is classified and assigned according to the classification standard of ecological suitability evaluation factors (Table 2). In the evaluation process, in order to reflect the principle of giving priority to ecological protection, firstly, ArcGIS software is used to conduct mosaic operation on the four indicators of ecological security factors: basic farmland protection, nature reserve, protected water area and cultural landscape to obtain the scope of the reserve; The four factors are substituted into formula (1) for weighted superposition operation to obtain the ecological security factor map—use the other index layers of exaction in the scope of the reserve and substitute other indexes into formula (2) for weighted superposition operation to obtain the natural and social factor map—then mosaically add the ecological security factor map and the natural and social factor map to obtain the comprehensive suitability evaluation value of regional construction land in mountainous villages and towns with multifactor weighted superposition [16]. Using *k*-means clustering method, it is divided into five categories: the most suitable land, more suitable land, basically suitable land, unsuitable land, and unavailable land. Finally, it is reclassified according to the suitability rating system of construction land (Table 1), the unsuitable land and unavailable land are divided into basic ecological control areas, the most suitable land and more suitable land are divided into construction control areas, and the basic suitable land is listed as ecological buffer areas. Using the classification results output by ArcGIS, the basic ecological control area determined by the model method is basically consistent with the current basic ecological control line of a city, indicating that the model is practical and scientific [17, 18].

## 5. Conclusion

Land suitability evaluation based on GIS has gone through great strides from the beginning to now, from simple superposition analysis to comprehensive analysis of multiple evaluation factors, and then to the application of more comprehensive methods such as artificial intelligence. In the evaluation analysis, the quantification of evaluation indexes and how to apply GIS to the whole decision-making process are the most critical parts. The weight of each evaluation index is determined by analytic hierarchy process, which reduces the subjectivity of weight evaluation. The multifactor comprehensive evaluation model is used to evaluate the ecological suitability of regional construction land in mountainous villages and towns. On this basis, combined with the actual situation, the basic ecological control area and construction control area are divided, and the suggestions on land use in mountainous villages and towns are put forward from the perspective of protecting the ecological security of mountainous villages and towns. It is of great significance for the scientific evaluation of the regional construction land of mountainous villages and towns and the development of mountainous villages and towns in the future. The role of GIS in the whole evaluation process has been constantly updated and improved, from single to open. There are some technical problems in the development of GIS, such as accuracy and expressiveness.

## Figures and Tables

**Figure 1:** Ecological suitability evaluation system of urban construction land.

**Figure 2:** Average random consistency index.

**Table 1:** Suitability grade system of construction land.

Suitable grade	Grade description	Division of construction area	Division of ecological control
Most suitable	Priority should be given to construction land	Suitable construction area	Construction control area
More suitable	Suitable for construction land		
Basically suitable	As a construction land, the effect is not obvious		Ecological buffer zone
Unsuitable	Generally, it is not used as construction land	Restricted area	Basic ecological control area
Unavailable land	It cannot be used as construction land	Forbidden area	

**Table 2:** Total ranking of evaluation index weights.

	Natural factor *B*1	Socio economic factors *B*2	Ecological security factor *B*3	
	0.2325	0.1396	0.5278	Total ranking weight of layer *C*
Elevation *C*1	0.1153	0	0	0.071589
Slope *C*2	0.2083	0	0	0.049326
Slope direction *C*3	0.0644	0	0	0.014088
Geomorphic type *C*4	0.1586	0	0	0.025902
Foundation bearing capacity *C*5	0.1175	0	0	0.039002
River *C*6	0.0579	0	0	0.019259
Lakes, reservoirs and sea areas *C*7	0.0258	0	0	0.024219
Vegetation *C*8	0.1306	0	0	0.043491
Land use status *C*9	0	0.1069	0	0.014923
Built up area *C*10	0	0.4862	0	0.047987
National and provincial highway *C*11	0	0.2845	0	0.053494
County road and township road *C*12	0	0.1789	0	0.023481
Basic farmland protection *C*13	0	0	0.0987	0.057425
Nature reserve *C*14	0	0	0.4156	0.216398
Protected waters *C*15	0	0	0.2895	0.142137
Cultural landscape *C*16	0	0	0.1938	0.011841

## Data Availability

The data used to support the findings of this study are available from the corresponding author upon request.
